# The role of acute care surgeons in treating rib fractures—a retrospective cohort study from a single level I trauma center

This article has been retracted.

**DOI:** 10.1186/s12893-022-01720-x

**Published:** 2022-07-14

**Authors:** Chia-Cheng Wang, Szu-An Chen, Chi-Tung Cheng, Yu-San Tee, Sheng-Yu Chan, Chih-Yuan Fu, Chien-An Liao, Chi-Hsun Hsieh, Ling-Wei Kuo

**Affiliations:** Department of Trauma and Emergency Surgery, Chang Gung Memorial Hospital, Linkou Medical Center, No. 5, Fuxing St., Guishan District, Taoyuan, 333 Taiwan

**Keywords:** Rib fracture, Acute care surgery, Surgical stabilization of rib fractures, SSRF, Trauma

## Abstract

**Background:**

Rib fractures are the most common thoracic injury in patients who sustained blunt trauma, and potentially life-threatening associated injuries are prevalent. Multi-disciplinary work-up is crucial to achieving a comprehensive understanding of these patients. The present study demonstrated the experience of an acute care surgery (ACS) model for rib fracture management from a single level I trauma center over 13 years.

**Methods:**

Data from patients diagnosed with acute rib fractures from January 2008 to December 2020 were collected from the trauma registry of Chang Gung Memorial Hospital (CGMH). Information, including patient age, sex, injury mechanism, Abbreviated Injury Scale (AIS) in different anatomic regions, injury severity score (ISS), index admission department, intensive care unit (ICU) length of stay (LOS), total admission LOS, mortality, and other characteristics of multiple rib fracture, were analyzed. Patients who received surgical stabilization of rib fractures (SSRF) were analyzed separately, and basic demographics and clinical outcomes were compared between acute care and thoracic surgeons.

**Results:**

A total of 5103 patients diagnosed with acute rib fracture were admitted via the emergency department (ED) of CGMH in the 13-year study period. The Department of Trauma and Emergency Surgery (TR) received the most patients (70.8%), and the Department of Cardiovascular and Thoracic Surgery (CTS) received only 3.1% of the total patients. SSRF was initiated in 2017, and TR performed fixation for 141 patients, while CTS operated for 16 patients. The basic demographics were similar between the two groups, and no significant differences were noted in the outcomes, including LOS, LCU LOS, length of indwelling chest tube, or complications. There was only one mortality in all SSRF patients, and the patient was from the CTS group.

**Conclusions:**

Acute care surgeons provided good-quality care to rib fracture patients, whether SSRF or non-SSRF. Acute care surgeons also safely performed SSRF. Therefore, we propose that the ACS model may be an option for rib fracture management, depending on the deployment of staff in each institute.

## Introduction

Trauma surgeons frequently encounter chest trauma. Approximately 40% of patients with an injury severity score (ISS) greater than 16 had concomitant thoracic injuries in Taiwan [1], and these injuries are accountable for up to 25% of trauma deaths [2]. Rib fractures are the most common thoracic injury in patients who sustained blunt trauma, and associated injuries with potential life-threatening outcomes often occur in these patients [3]. Contrary to common perception, rib fractures should not be taken lightly. Patients suffering from motor vehicle collisions with rib fractures have a 4.4% 30 day mortality rate, and mortality increases with the greater the number of fractured ribs [4].

Surgical stabilization of rib fractures (SSRF) has gained substantial popularity as a treatment option in the past decade. Previous studies revealed that SSRF benefitted patients with flail chest [5], non-flail displaced fractures [6], and patients who were ventilator-dependent [7]. Although SSRF is generally considered an operation by thoracic surgeons, other subspecialties, including orthopedic surgeons, general surgeons, and acute care trauma surgeons, are deeply involved in the treatment of rib fractures and SSRF [8–10].

Several factors influence the outcomes of patients undergoing SSRF, including time and experience of the facility [11], the timing of surgery [12], injury severity, and the variation in hospital levels [13]. However, whether the subspecialty of the treating surgeon is also an essential factor is not clear. The present study analyzed the pattern and outcomes of rib fractures and SSRF between cardiovascular and thoracic surgeons and acute care surgeons and discussed the preliminary outcome of the acute care surgery (ACS) model for rib fracture patients.

## Materials and methods

The present study was a retrospective cohort study. Data were extracted from the trauma registry of Chang Gung Memorial Hospital (CGMH). CGMH is a level 1 trauma center with 3700 beds that serves as a major trauma referral hospital for northern Taiwan. At least two to three acute care trauma team attending surgeons remain in-house, and all of the subspecialties are available for consultation 24/7. Trauma patients with a diagnosis of rib fracture in all age groups and injury severities who presented to the emergency department (ED) of CGMH from Jan 1, 2008 to Dec 31, 2020 were included in this study. All trauma patients were managed under Advanced Trauma Life Support (ATLS) guidelines. After the primary survey and/or secondary survey in the ED, patients were admitted to the corresponding department according to their primary diagnosis that needed the most immediate attention. Subspecialty consultation and discussion was coordinated by the in-house acute care surgeon when multiple injuries occurred. If no agreement between subspecialties was reached in the admitting department, the patient was admitted to the Department of Trauma and Emergency Surgery. SSRF was first introduced to CGMH in 2017. Before our first SSRF, rib fracture patients were treated using a conservative approach centered on pain control and respiratory rehabilitation (Fig. 1a). SSRF has been integrated into our standard treatment protocol since 2017 (Fig. 1b). Only acute rib fracture patients who entered the ED were enrolled in this study. Patients with subacute or chronic rib fractures treated and admitted via outpatient clinics were excluded from the analysis.

**Fig. 1:** The treatment protocol for rib fracture patients in CGMH. **a** Standard treatment prior to SSRF. **b** The treatment algorithm for SSRF

Structural analysis was performed for all patients, regardless of SSRF. Basic demographics, including age, sex, severity, and crude outcomes of each subspecialty, were compared using the chi-squared test and Kruskal–Wallis test, as appropriate. The subspecialties included the Department of Trauma and Emergency Surgery (TR), the Department of Cardiovascular and Thoracic Surgery (CTS), the Department of Neurosurgery (NS), the Department of Plastic and Reconstruction Surgery (PS), the Department of Orthopedic Surgery (Ortho), and other miscellaneous departments. The same approach was used for patients with ISS ≥ 16 and ISS ≥ 25 to examine whether there was an architectural difference as injury severity escalated. For surgically treated patients, we compared the two subspecialties involved in SSRF (TR and CTS). Basic demographics and outcomes, including length of stay, mortality, and complications, were analyzed using chi-squared and Mann–Whitney U tests. Due to an imbalanced patient number between the two departments, a propensity-score matching analysis was performed to eliminate potential bias. We performed the statistical analyses using IBM SPSS Statistics for Windows V.22.0 (IBM Corp., Armonk, NY).

## Results

A total of 5103 patients diagnosed with acute rib fracture were admitted via the ED of CGMH in the 13-year study period. TR, CTS, and NS received patients with higher ISS, and patients of PS and Ortho were in less critical condition. Greater than 70% of these patients were treated by TR, and 14.7% were treated by NS. CTS primarily managed only 3.1% of the patients, but these patients had the most severe chest injuries, with a median chest abbreviated injury scale (AIS) of 4 (Table 1a). Similar patterns were observed when we narrowed patients with ISS ≥ 16 (Table 1b) and ISS ≥ 25 (Table 1c). The overall mortality rates of all patients for TR, CTS, and NS were 3.0%, 11.5%, and 13.9%, respectively, and the rate increased as severity escalated. However, TR still had relatively lower mortality numbers in the ISS ≥ 16 and ISS ≥ 25 groups, despite narrowing the margin of ISS.

**Table 1:** Crude analysis for all rib fracture patients

Variables	Total (n = 5103)						P value
	TR (n = 3611, 70.8%)	CTS (n = 156, 3.1%)	NS (n = 750, 14.7%)	PS (n = 76, 1.5%)	Ortho (n = 489, 9.6%)	Other (n = 21, 0.4%)	
a. Distribution, basic demographics, and outcomes for all rib fracture patients							
Sex (male, ratio)	2606 (72.2%)	135 (86.5%)	536 (71.5%)	56 (73.7%)	329 (67.3%)	13 (61.9%)	< 0.001
Age (Median, IQR)	54 (40–65)	47.5 (33–58)	55 (43–67)	47 (31–59)	53 (38–64)	53 (14–71)	< 0.001
ISS (Median, IQR)	16 (10–24)	21 (16–29)	29 (20–36)	13 (9–22)	13 (8–18)	14 (10–22)	< 0.001
Chest AIS (Median, IQR)	3 (3–4)	4 (4–4)	3 (2–4)	2 (1–3)	2 (1–3)	3 (2–4)	< 0.001
NISS (Median, IQR)	18 (13–27)	29 (18–36)	30 (22–41)	15.5 (11–23)	14 (10–22)	16 (10–29)	< 0.001
ICU LOS (Median, IQR)	0 (0–4)	4 (2–7)	3 (0–9)	0 (0–6)	0 (0–0)	2 (0–3)	< 0.001
Total LOS (Median, IQR)	9 (5–15)	13 (7–19)	13 (6–25)	13.5 (6.5–20.5)	9 (6–15)	6 (4–14)	< 0.001
Mortality (ratio)	107 (3.0%)	18 (11.5%)	104 (13.9%)	2 (2.6%)	3 (0.6%)	2 (9.5%)	< 0.001

Variables	Total (n = 3040)						P value
	TR (n = 2044, 67.2%)	CTS (n = 131, 4.3%)	NS (n = 672, 22.1%)	PS (n = 32, 1.1%)	Ortho (n = 151, 5.0%)	Other (n = 10, 0.3%)	
b. Distribution, basic demographics, and outcomes for all rib fracture patients with ISS ≥ 16							
Sex (male, ratio)	1516 (74.2%)	113 (86.3%)	488 (72.6%)	23 (71.9%)	105 (69.5%)	5 (50%)	0.008
Age (Median, IQR)	51 (38–63)	47 (31–59)	55 (42–67)	45 (21–62)	50 (35–62)	42 (14–68)	< 0.001
ISS (Median, IQR)	22 (19–29)	24 (20–29)	29 (24–36)	22 (18–29)	22 (18–25)	24 (21–32)	< 0.001
Chest AIS (Median, IQR)	4 (3–4)	4 (4–4)	3 (2–4)	3 (2–3)	3 (3–4)	4 (3–4)	< 0.001
NISS (Median, IQR)	25 (20–34)	29 (24–41)	34 (24–41)	24 (22–29)	27 (22–29)	31 (21–36)	< 0.001
ICU LOS (Median, IQR)	3 (0–6)	5 (2–8)	4 (0–10)	4.5 (0–11)	0 (0–4)	2 (0–4)	< 0.001
Total LOS (Median, IQR)	12 (8–20)	15 (9–22)	14 (7–26)	18.5 (14–29.5)	15 (10–22)	6.5 (3–16)	< 0.001
Mortality (ratio)	101 (4.9%)	18 (13.7%)	104 (15.5%)	2 (6.3%)	3 (2.0%)	2 (20%)	0.002

Variables	Total (n = 1464)						P value
	TR (n = 867, 59.2%)	CTS (n = 64, 4.4%)	NS (n = 462, 31.6%)	PS (n = 9, 0.6%)	Ortho (n = 57, 3.9%)	Other (n = 5, 0.3%)	
c. Distribution, basic demographics, and outcomes for all rib fracture patients with ISS ≥ 25							
Sex (male, ratio)	651 (75.1%)	56 (87.5%)	348 (75.3%)	6 (66.7%)	37 (64.9%)	2 (40%)	0.034
Age (Median, IQR)	48 (34–61)	43 (31–55)	54.5 (42–67)	49 (20–61)	50 (36–60)	14 (14–40)	< 0.001
ISS (Median, IQR)	32 (29–36)	29 (26–34)	34 (29–38)	29 (29–33)	27 (25–34)	32 (29–34)	< 0.001
Chest AIS (Median, IQR)	4 (3–4)	4 (4–5)	3 (3–4)	4 (2–4)	4 (3–4)	3 (3–4)	< 0.001
NISS (Median, IQR)	34 (29–41)	41 (34–43)	38 (33–43)	34 (29–38)	33 (29–34)	34 (32–45)	< 0.001
ICU LOS (Median, IQR)	5 (3–11)	6.5 (4–11)	6 (2–12)	2 (0–7)	3 (0–6)	2 (2–4)	0.002
Total LOS (Median, IQR)	17 (11–26)	18 (11.5–27)	19 (9–29)	22 (13–29)	18 (13–28)	9 (2–16)	0.360
Mortality (ratio)	84 (9.7%)	15 (23.4%)	98 (21.2%)	2 (22.2%)	2 (3.5%)	1 (20%)	0.428

*ISS* injury severity score, *AIS* Abbreviated Injury Scale, *NISS* new injury severity score, *ICU* intensive care unit, *LOS* length of stay

One hundred fifty-seven patients received SSRF in the study period. TR was performed on 141 patients, and only 16 patients received SSRF by CTS (Table 2). There were no significant differences in basic demographics for the patients operated by TR or CTS in the gross comparison. Chest AIS, ISS, and the New ISS (NISS) appeared higher in CTS patients, but none of the differences reached statistical significance. The complication rate was higher in the CTS group (31.3% vs. 12.8%, p = 0.048), and mortality was present in only CTS patients. Due to the wide gap in patient numbers, propensity score matching (PSM) with a matching ratio of 1:4 was performed to eliminate potential bias from the inequality of patient volume. The significance of complications disappeared in the outcome analysis after PSM (Table 3), except for the p value of mortality rate, which remained under 0.05. However, one death out of 16 patients might not clinically meaningful.

**Table 2:** Comparison of outcomes between TR and CTS patients

Variables	Total Patients Received SSRF (n = 157)		
	TR (n = 141)	CTS (n = 16)	P value
Age (Median, IQR)	56 (49–67)	57.5 (48.5–63.5)	0.796
Sex (Male, ratio)	45 (31.9%)	6 (37.5%	0.651
Flail chest (ratio)	79 (56.0%)	8 (50%)	0.646
Numbers of Fractured Ribs (Median, IQR)	6 (5–8)	6 (4.5–9.5)	0.883
Numbers of Fractures (Median, IQR)	8 (5–11)	8 (4.5–12.5)	0.958
Chest AIS (Median, IQR)	3 (2–4)	3.5 (1–4)	0.374
ISS (Median, IQR)	20 (16–29)	23.5 (23.5)	0.411
NISS (Median, IQR)	24 (17–33)	32.5 (22–39.5)	0.094
Total LOS (Median, IQR)	13 (10–16)	17 (10.5–26.5)	0.095
ICU LOS (Median, IQR)	0 (0–5)	3 (0–6.5)	0.324
Length of MV (Median, IQR)	0 (0–2)	1.5 (0–4)	0.193
Length of CT (Days, median, IQR)	8 (5–11)	10 (3.5–16)	0.787
Complication (ratio)	18 (12.8%)	5 (31.3%)	0.048
Mortality (ratio)	0 (0%)	1 (6.3%)	0.003

*ISS* injury severity score, *AIS* Abbreviated Injury Scale, *NISS *new injury severity score, *ICU *intensive care unit, *LOS* length of stay, *MV* mechanical ventilation, *CT*  chest tube, *TR*  Department of Trauma and Emergency Surgery, *CTS* Department of Cardiovascular and Thoracic Surgery

**Table 3:** Comparison of outcomes between TR and CTS patients after propensity score matching

Variables	Outcome analysis after PSM		
	TR (n = 64)	CTS (n = 16)	P value
Total LOS (Median, IQR)	14 (11–18)	17 (10.5–26.5)	0.049
ICU LOS (Median, IQR)	2 (0–8)	3 (0–6.5)	0.867
Length of MV (Median, IQR)	0 (0–3)	1.5 (0–4)	0.537
Length of CT (Median, IQR)	9 (6–13)	10 (3.5–16)	0.867
Complication	10	5	0.152
Mortality	0	1	0.044

*ICU* intensive care unit, *LOS* length of stay, *MV* mechanical ventilation, *CT* chest tube, *TR* Department of Trauma and Emergency Surgery, *CTS* Department of Cardiovascular and Thoracic Surgery

More detailed descriptions of the complications are listed in Table 4. Twenty-three patients experienced complications, 18 in TR and 5 in CTS. Four patients (3 in the TR group and 1 in the CTS group) experienced hardware failure, including screw dislodgement and plate fracture. Notably, all 3 failures in the TR group occurred before 2019. Prolonged opioid use was defined as the need for intravenous or oral opioid use one month after the surgery due to the increased risk of long-term opioid use [14]. Two patients in the TR group presented with this condition, but none of the CTS patients had this adverse effect. Pulmonary complications occurred in 18 TR patients and 4 CTS patients, and one CTS patient developed concomitant post-operative pneumonia and empyema. None of the patients suffered from malunion, but three patients in the TR group suffered from non-fracture-related adverse events (2 ischemic strokes and one intracranial hemorrhage).

**Table 4:** List of complications

Variables	Total complications (n = 23)	
	TR (n = 18)	CTS (n = 6)
Sugery/ implant related	6	2
Hardware failure	3	1
Wound infection	1	0
Prolong opioid use	2	0
Bone healing	0	0
Pulmonary	9	4
Pneumonia	7	3
Empyema	1	1
Residual pneumothorax	1	1
Other	3	0
Ischemic stroke	2	0
I ntracranial hemorrhage	1	0

*TR* Department of Trauma and Emergency Surgery, *CTS* Department of Cardiovascular and Thoracic Surgery

## Discussion

Treatment outcomes and subspecialization were discussed in various clinical practice fields, including surgical or medical. Treatment by subspecialty clinicians shared excellent benefits in some studies [15, 16], but the benefit of subspecialization may be marginal in some aspects [17, 18]. The management of trauma and acute care surgery is an emerging subspecialty, but it requires a great deal of generalization. A trauma surgeon should focus on anatomy, pathology, the patient's physiology and rearrangement of impaired physiology [19]. Using rib fractures as an example, injuries to at least three body regions were found in as many as 60% of patients with rib fractures [20], and solid organ injuries below the diaphragm are very common concomitant findings in these patients [21]. Therefore, treatment for these patients requires attention to intra-thoracic complications and diagnosis and the management of extra-thoracic injuries.

Our dataset disclosed that the acute care trauma team treated most patients with rib fractures, regardless of severity, in CGMH for more than a decade, and we generated substantial outcomes. One essential key is competence in general trauma management. Physicians perform better when they are trained and interested in a specific area than physicians who are not trained or have no particular interest in that area. As a result, surgeons committed to trauma outperform with fewer missed injuries than surgeons in other subspecialties [22]. Another pillar to maintaining our trauma care system is the continuity of care. Having at least 2 to 3 in-house attending surgeons 24/7 provides several benefits to patients. Timely treatment is an important rule for severely injured patients. Van der Vliet reported that in-house trauma surgeons shortened the time from ED to ICU and ED to surgery to nearly 50% [23]. Care quality is also crucial after stabilizing trauma patients. Management continuity is fundamental in complex clinical diseases that require management from several providers who potentially work at cross purposes [24]. With multiple in-house attending surgeons, the quality is continued day or night, weekdays or holidays, or different levels of duty residents.

Another decisive factor is the team attitude toward involvement with rib fractures and thoracic trauma, as surgeons’ attitudes toward certain trauma scenarios differ [25], and skill sets can also vary between individuals and facilities [26]. Therefore, the willingness to take care of a new patient group is crucial for developing competency. Doubts in self-efficacy can be a large barrier that prevent physicians from carrying out proper treatment for their patients [27], and only when the whole team is devoted can we form a consensus on how to manage patients with rib fractures and further improve the quality of care. It is also very important that our institute has been very generous in investing resources in the field of trauma treatment, and this level of commitment could result in overall improved outcomes [28]. In sum, the acute care surgeons in our institute showed great interest in taking care of a large volume of complicated trauma patients since day one, which was long before SSRF was introduced, and our working system ensured the promptness of care, which resulted in good quality of care, as demonstrated in our data.

The TR team was also the first group in our institute to introduce this procedure for treating acutely injured patients with rib fractures in the SSRF era. Video-assisted thoracic surgery (VATS) plays a significant role in SSRF. Although not yet considered necessary as a routine approach [29], evacuating hemothoraces and proper chest tube placement are crucial for SSRF, especially when the pleural space is violated [30]. Stereotypical thinking suggests that acute care surgeons are not familiar with the VATS approach. While VATS may not be a universal approach for all acute care surgeons, multiple studies have shown that acute care surgeons can perform this procedure safely and effectively [31, 32]. Our data supported this concept as they show similar outcomes and complication rates (Table 4) as previous studies [33]. The lack of hardware failure after 2019 shows that as experience accumulated and surgeons became more familiar with the prostheses and instruments, preventable complications could be avoided. Previous studies have shown that surgeon experience reduces hardware failure rates in orthopedic procedures [34,35], and our results are consistent with this evidence, which indicates that patient volume may play a more prominent role than subspecialties in this issue.

The comparison between TR and CTS may be statistically flawed because the patient numbers were heavily tilted to one side. However, the main goal of the present study was to describe that non-inferiority could be achieved by an acute care surgery (ACS) model for rib fracture patients not to prove that acute care surgeons could outperform thoracic surgeons. Acute care surgeons should not replace certain subspecialties, but the system should be reinvented to introduce more comprehensive care to the patients. The ACS model is beneficial for some general surgery diseases, such as acute appendicitis [36] or gallstone pancreatitis[37], and a similar model would be advantageous for rib fractures, regardless of whether SSRF is indicated in each patient. Considerable evidence revealed that the ACS model separated emergent and elective surgery groups and improved staff efficiency to increase revenue for the emergent and elective surgery groups [38, 39]. The treatment for rib fractures can develop a similar pattern via the management of most patients by acute care surgeons, which leaves a small portion of complicated cases to the expert thoracic surgeons. Therefore, thoracic surgeons could focus on elective surgeries and eventually generate maximal efficiency and productivity for both teams.

There are some limitations to this study. This study was a single-institute study with only four years of SSRF experience. The long-term results of the ACS model must be confirmed in future studies. The retrospective nature of our analysis is another shortcoming, which may pose potential bias. Ideally, more parameters should be involved in the investigation, e.g., pain scales, lung function tests, and daily activities. A well-designed prospective study will provide more information and enable a more thorough understanding of accurate patient outcomes. The effect of the learning curves of individual surgeons was not included in the present study, but a more senior surgeon often performed a joint operation with a less experienced surgeon in our routine practice. Therefore, the potential influence may be diluted and difficult to demonstrate. Lastly, the results of our institute may not be reproducible in other hospitals, especially when the ACS model is not mature.

## Conclusion

Acute care surgeons provide good-quality care to rib fracture patients, whether SSRF or non-SSRF. The ACS model offers several advantages, including comprehensive care for poly-trauma, avoiding missed injuries, and timely decision-making and treatment. Acute care surgeons may safely perform SSRF. Therefore, we propose the ACS model as an option for rib fracture management, depending on the deployment of staff in each institute.

## Data Availability

The data that support the findings of this study are available from the CGMH trauma registry, but restrictions apply to the availability of these data, which were used under license for the current study and are not publicly available. However, data are available from the authors upon reasonable request and with permission of the Chang Gung Medical Foundation Institutional Review Board and the CGMH trauma registry.

## Abbreviations

ACS: Acute care surgery
CGMH: Chang Gung Memorial Hospital
AIS: Abbreviated injury scale
ISS: Injury severity score
NISS: New injury severity score
ICU: Intensive care unit
LOS: Length of stay
SSRF: Surgical stabilization of rib fractures
ED: Emergency department
TR: Department of Trauma and Emergency Surgery
CTS: Department of Cardiovascular and Thoracic Surgery
NS: Department of Neurosurgery
PS: Department of Plastic and Reconstruction Surgery
Ortho: Department of Orthopedic Surgery
PSM: Propensity score matching
VATS: Video-Assisted Thoracic Surgery

## References

[1] Kuo LW, Fu CY, Liao CA, Liao CH, Hsieh CH, Wang SY (2019). Inequality of trauma care under a single-payer universal coverage system in Taiwan: a nationwide cohort study from the National Health Insurance Research Database. BMJ Open.

[2] Lin FC, Li RY, Tung YW, Jeng KC, Tsai SC (2016). Morbidity, mortality, associated injuries, and management of traumatic rib fractures. J Chin Med Assoc.

[3] Brasel KJ, Moore EE, Albrecht RA, deMoya M, Schreiber M, Karmy-Jones R (2017). Western trauma association critical decisions in trauma: management of rib fractures. J Trauma Acute Care Surg.

[4] Lien Y-C, Chen C-H, Lin H-C (2009). Risk factors for 24-hour mortality after traumatic rib fractures owing to motor vehicle accidents: a nationwide population-based study. Ann Thorac Surg.

[5] Leinicke JA, Elmore L, Freeman BD, Colditz GA (2013). Operative management of rib fractures in the setting of flail chest: a systematic review and meta-analysis. Ann Surg.

[6] Pieracci FM, Leasia K, Bauman Z, Eriksson EA, Lottenberg L, Majercik S (2020). A multicenter, prospective, controlled clinical trial of surgical stabilization of rib fractures in patients with severe, nonflail fracture patterns (Chest Wall Injury Society NONFLAIL). J Trauma Acute Care Surg.

[7] Wada T, Yasunaga H, Inokuchi R, Matsui H, Matsubara T, Ueda Y (2015). Effectiveness of surgical rib fixation on prolonged mechanical ventilation in patients with traumatic rib fractures: a propensity score-matched analysis. J Crit Care.

[8] Mayberry JC, Ham LB, Schipper PH, Ellis TJ, Mullins RJ (2009). Surveyed opinion of American trauma, orthopedic, and thoracic surgeons on rib and sternal fracture repair. J Trauma.

[9] Sarani B, Allen R, Pieracci FM, Doben AR, Eriksson E, Bauman ZM (2019). Characteristics of hardware failure in patients undergoing surgical stabilization of rib fractures: A Chest Wall Injury Society multicenter study. J Trauma Acute Care Surg.

[10] Minervini F, Kestenholz PB, Bertoglio P, Scarci M, Kocher GJ (2020). Surgical management of rib fractures in chest wall trauma. J Visc Surg.

[11] Prins JTH, Leasia K, Sauaia A, Burlew CC, Cohen MJ, Coleman JJ (2021). A decade of surgical stabilization of rib fractures: the effect of study year on patient selection, operative characteristics, and in-hospital outcome. Injury.

[12] Chen Zhu R, de Roulet A, Ogami T, Khariton K (2020). Rib fixation in geriatric trauma: Mortality benefits for the most vulnerable patients. J Trauma Acute Care Surg.

[13] Kane ED, Jeremitsky E, Pieracci FM, Majercik S, Doben AR (2017). Quantifying and exploring the recent national increase in surgical stabilization of rib fractures. J Trauma Acute Care Surg.

[14] Shah A, Hayes CJ, Martin BC (2017). Characteristics of initial prescription episodes and likelihood of long-term opioid use—United States, 2006–2015. MMWR Morb Mortal Wkly Rep.

[15] du Bois A, Rochon J, Pfisterer J, Hoskins WJ (2009). Variations in institutional infrastructure, physician specialization and experience, and outcome in ovarian cancer: a systematic review. Gynecol Oncol.

[16] Johannson KA, Lethebe BC, Assayag D, Fisher JH, Kolb M, Morisset J (2022). Travel distance to subspecialty clinic and outcomes in patients with fibrotic interstitial lung disease. Ann Am Thorac Soc.

[17] Schumaier AP, Andrews EG, Yue RA, Lake SS, Evans HT, Scarberry NW (2020). Hemiarthroplasty for femoral neck fractures: does surgeon subspecialty affect perioperative outcomes?. J Orthop Trauma.

[18] Mielke D, Malinova V, Moerer O, Suntheim P, Voit M, Rohde V (2019). Does the subspecialty of an intensive care unit (ICU) has an impact on outcome in patients suffering from aneurysmal subarachnoid hemorrhage?. Neurosurg Rev.

[19] Kurihara H (2017). Acute care surgery: a necessity across Europe. Are we ready to take the lead?. Chirurgia.

[20] Caragounis EC, Xiao Y, Granhed H (2021). Mechanism of injury, injury patterns and associated injuries in patients operated for chest wall trauma. Eur J Trauma Emerg Surg.

[21] Kessel B, Dagan J, Swaid F, Ashkenazi I, Olsha O, Peleg K (2014). Rib fractures: comparison of associated injuries between pediatric and adult population. Am J Surg.

[22] Lin Y-K, Lin C-J, Chan H-M, Lee W-C, Chen C-W, Lin H-L (2014). Surgeon commitment to trauma care decreases missed injuries. Injury.

[23] van der Vliet QMJ, van Maarseveen OEC, Smeeing DPJ, Houwert RM, van Wessem KJP, Simmermacher RKJ (2019). Severely injured patients benefit from in-house attending trauma surgeons. Injury.

[24] Haggerty JL, Reid RJ, Freeman GK, Starfield BH, Adair CE, McKendry R (2003). Continuity of care: a multidisciplinary review. BMJ.

[25] Manson J, Burke K, Starnes CP, Long K, Kearney PA, Bernard A. Paramedic and Surgeon Views on Trauma Surgical Readiness: Implications for Guideline Implementation. Am Surg. 2018;84(6):1079–85.29981652

[26] Cothren CC, Moore EE, Hoyt DB. The U.S. trauma surgeon’s current scope of practice: can we deliver acute care surgery? J Trauma. 2008;64(4):955–65; discussion 965-8.10.1097/TA.0b013e318169214818404062

[27] Cabana MD, Rand CS, Powe NR, Wu AW, Wilson MH, Abboud PA, et al. Why don’t physicians follow clinical practice guidelines? A framework for improvement. JAMA. 1999;282(15):1458–65.10.1001/jama.282.15.145810535437

[28] Mains C, Scarborough K, Bar-Or R, Hawkes A, Huber J, Bourg P, et al. Staff commitment to trauma care improves mortality and length of stay at a level I trauma center. J Trauma. 2009;66(5):1315–20.10.1097/TA.0b013e31819d96d819430233

[29] Bui JT, Browder SE, Wilson HK, Kindell DG, Ra JH, Haithcock BE, et al. Does routine uniportal thoracoscopy during rib fixation identify more injuries and impact outcomes? J Thorac Dis. 2020;12(10):5281–8.10.21037/jtd-20-2087PMC765641033209362

[30] Pieracci FM, Majercik S, Ali-Osman F, Ang D, Doben A, Edwards JG, et al. Consensus statement: Surgical stabilization of rib fractures rib fracture colloquium clinical practice guidelines. Injury. 2017;48(2):307–21.10.1016/j.injury.2016.11.02627912931

[31] Smith JW, Franklin GA, Harbrecht BG, Richardson JD. Early VATS for blunt chest trauma: a management technique underutilized by acute care surgeons. J Trauma. 2011;71(1):102–5; discussion 105-7.10.1097/TA.0b013e318222308021818019

[32] Pottenger BC, Galante JM, Wisner DH. The modern acute care surgeon: characterization of an evolving surgical niche. J Trauma Acute Care Surg. 2015;78(1):120–5.10.1097/TA.000000000000049625539212

[33] Peek J, Beks RB, Hietbrink F, Heng M, De Jong MB, Beeres FJP, et al. Complications and outcome after rib fracture fixation: A systematic review. J Trauma Acute Care Surg. 2020;89(2):411–8.10.1097/TA.000000000000271632282759

[34] Haskell A, Mann RA. Perioperative complication rate of total ankle replacement is reduced by surgeon experience. Foot Ankle Int. 2004;25(5):283–9.10.1177/10711007040250050215134607

[35] Ward CM, Kuhl TL, Adams BD. Early complications of volar plating of distal radius fractures and their relationship to surgeon experience. Hand . 2011;6(2):185–9.10.1007/s11552-010-9313-5PMC309288822654702

[36] Fu CY, Huang HC, Chen RJ, Tsuo HC, Tung HJ (2014). Implementation of the acute care surgery model provides benefits in the surgical treatment of the acute appendicitis. Am J Surg.

[37] Murphy PB, Paskar D, Hilsden R, Koichopolos J, Mele TS (2017). Acute care surgery: a means for providing cost-effective quality care for gallstone pancreatitis. World J Emerg Surg..

[38] Barnes SL, Cooper CJ, Coughenour JP, MacIntyre AD, Kessel JW. Impact of acute care surgery to departmental productivity. J Trauma. 2011;71(4):1027–32; discussion 1033-4.10.1097/TA.0b013e318230714621986743

[39] Miller PR, Wildman EA, Chang MC, Meredith JW. Acute care surgery: impact on practice and economics of elective surgeons. J Am Coll Surg. 2012;214(4):531–5; discussion 536-8.10.1016/j.jamcollsurg.2011.12.04522397976

